The article "Matrine alleviates lipopolysaccharide-induced intestinal inflammation and oxidative stress via CCR7 signal" was retracted in 2023. Reasons: results that could not be reproduced; unreliable results or conclusions.

# Matrine alleviates lipopolysaccharide-induced intestinal inflammation and oxidative stress via CCR7 signal

**DOI:** 10.18632/oncotarget.14598

**Published:** 2017-01-11

**Authors:** Guojun Wu, Wenhong Zhou, Junfeng Zhao, Xiaohua Pan, Yongjie Sun, Hao Xu, Peng Shi, Chong Geng, Ling Gao, Xingsong Tian

**Affiliations:** ^1^ Department of Breast and Thyroid Surgery, Shandong Provincial Hospital Affiliated to Shandong University, Jinan 250021, Shandong, P. R. China; ^2^ Department of Nursing, Shandong Provincial Hospital Affiliated to Shandong University, Jinan 250021, Shandong, P. R. China; ^3^ Traffic Police Department, Jinan Public Security Bureau, Jinan 250021, Shandong, P. R. China; ^4^ Scientific Center, Shandong Provincial Hospital Affiliated to Shandong University, Jinan 250021, Shandong, P. R. China

**Keywords:** matrine, inflammation, oxidative stress, CCR7, LPS

## Abstract

The aim of this study was to investigate the protective effects of matrine on lipopolysaccharide (LPS)-induced inflammation and oxidative stress *in vivo* and *in vitro*. The results showed that matrine improved intestinal inflammatory status and oxidative balance and enhanced chemokine receptor 7 (CCR7) expression. In LPS-challenged mice and Caco-2 cells, matrine alleviated LPS-induced inflammation and oxidative stress via downregulating pro-inflammatory cytokines (IL-1β and IL-17) and malondialdehyde (MDA) production. CCR7-siRNA transfection blocked the protective effects of matrine on LPS-induced inflammation and oxidative stress and exacerbated LPS caused injury. In conclusion, matrine alleviates LPS-induced intestinal inflammation and oxidative stress in mice and Caco-2 cells, which may be associated with CCR7 signal.

## INTRODUCTION

Matrine, a quinolizidine alkaloid component of the Chinese herb, isolates from the roots of Sophora species, such as Sophora flavescens (Kushen), Sophora tonkinensis, and Sophora alopecuroides (Kudouzi) [1]. Various reports have suggested that matrine exhibits anti-inflammatory and antioxidant effects and may serve as a therapeutic potential for inflammation and oxidative stress relative diseases [2, 3]. For example, matrine alleviates cytokines production, inflammatory cell infiltration, and goblet cell differentiation by downregulating suppressor of cytokine signaling 3 and inhibiting nuclear factor kappa-B (NF-κB) signal in airway epithelial cells and asthmatic mice [4]. In the focal cerebral ischemic injury, matrine improves antioxidant activity via increasing antioxidant enzymes, such as superoxide dismutase (SOD), glutathione peroxidase (GSH-Px), and catalase (CAT) [5]. Furthermore, matrine and its derivatives have displayed anticancer activity, antiviral activity, analgesic effect, anti-fibrotic activity, insecticidal activity, and antimicrobial activity [1].

The article "Matrine alleviates lipopolysaccharide-induced intestinal inflammation and oxidative stress via CCR7 signal" was retracted in 2023. Reasons: results that could not be reproduced; unreliable results or conclusions.

Chemokine receptors (CCR) and their ligands play an important role in coordination of cell trafficking in many biological processes, especially for inflammation and oxidative stress [6]. However, there are little references about matrine and chemokine receptors mediated inflammation and oxidative stress. Thus, in this study, we used lipopolysaccharide (LPS) to induce inflammation and oxidative stress in mice and Caco-2 cells to investigate the protective role of matrine in LPS-induced inflammation and oxidative stress and the potential mechanism of chemokine receptors.

## RESULTS

### Matrine improves inflammatory status and antioxidant function in mice

Jejunal and ileal mRNA abundances IL-1β, IL-10, IL-17, and TNF-α were determined in this study (Table 1). In the jejunum, 10 mg/kg matrine significantly downregulated IL-1β expression compared with the control group (*P <* 0.05). In addition, matrine tended to influence IL-10 and TNF-α expression, while the difference was insignificant (*P >* 0.05). In the ileum, IL-1β was markedly lower in 10 mg/kg matrine group and IL-17 was downregulated in 5 and 10 mg/kg matrine groups compared with the control group (*P <* 0.05).

**Table 1:** Matrine improves inflammatory status in mice

Item	Control	1 mg/kg Matrine	5 mg/kg Matrine	10 mg/kg Matrine
Jejunum				
IL-1β	1.00 ± 0.11a	1.11 ± 0.13a	0.82 ± 0.14ab	0.76 ± 0.06b
IL-10	1.00 ± 0.17	1.03 ± 0.16	0.96 ± 0.11	0.75 ± 0.18
IL-17	1.00 ± 0.13	1.07 ± 0.11	1.03 ± 0.12	1.21 ± 0.15
TNF-α	1.00 ± 0.13	1.09 ± 0.15	1.05 ± 0.15	0.83 ± 0.14
Ileum				
IL-1β	1.00 ± 0.08a	0.96 ± 0.15a	1.08 ± 0.14a	0.73 ± 0.07b
IL-10	1.00 ± 0.11	0.89 ± 0.17	0.93 ± 0.14	1.06 ± 0.14
IL-17	1.00 ± 0.10ab	0.78 ± 0.16ab	0.77 ± 0.08b	0.69 ± 0.05b
TNF-α	1.00 ± 0.13	1.05 ± 0.07	0.91 ± 0.11	0.88 ± 0.18

Data are expressed as the mean ± standard error of the mean. Values in the same row with different superscripts are significant (*P <* 0.05), while values with same superscripts are not significant different (*P* > 0.05).

SOD, total antioxidant capacity (T-AOC), and malondialdehyde (MDA) have been widely served as oxidative makers. In this study, we found that dietary matrine (5 and 10 mg/kg) significantly enhanced jejunal and ileal T-AOC activities and MDA abundance was marked lower in 10 mg/kg matrine group than that in the control group (*P <* 0.05) (Table 2).

**Table 2:** Matrine improves intestinal antioxidant function in mice

Item	Control	1 mg/kg Matrine	5 mg/kg Matrine	10 mg/kg Matrine
Jejunum				
SOD U/mgprot	84.23 ± 7.23	88.26 ± 11.29	82.92 ± 14.15	96.27 ± 12.03
T-AOC U/gprot	0.57 ± 0.07b	0.61 ± 0.07b	0.93 ± 0.12a	1.12 ± 0.14a
MDA uM/mgprot	11.69 ± 1.13a	10.02 ± 1.83ab	10.24 ± 1.27ab	8.51 ± 0.82b
Ileum				
SOD U/mgprot	78.28 ± 10.17	96.23 ± 15.18	86.07 ± 14.73	91.74 ± 9.18
T-AOC U/gprot	0.56 ± 0.07	0.63 ± 0.07b	0.86 ± 0.11a	0.93 ± 0.12a
MDA uM/mgprot	18.42 ± 2.46a	16.52 ± 2.84a	15.27 ± 2.27ab	13.93 ± 1.32b

Data are expressed as the mean ± standard error of the mean. Values in the same row with different superscripts are significant (*P <* 0.05), while values with same superscripts are not significant different (*P* > 0.05).

The article "Matrine alleviates lipopolysaccharide-induced intestinal inflammation and oxidative stress via CCR7 signal" was retracted in 2023. Reasons: results that could not be reproduced; unreliable results or conclusions.

### Matrine activates intestinal chemokine receptors in mice

Chemokine receptors are widely involved in inflammatory response, thus intestinal expressions of CCR2, CCR5, CCR6, CCR7, and CCR7 were tested (Table 3). In the jejunum, 5 mg/kg matrine enhanced CCR7 expression and 10 mg/kg matrine markedly upregulated CCR5, CCR6, and CCR7 expressions compared with the control group (*P <* 0.05). In the ileum, dietary matrine (1, 5, and 10 mg/kg) increased CCR7 mRNA level and 10 mg/kg matrine markedly enhanced CCR2, CCR5, and CCR7 expressions (*P <* 0.05).

**Table 3:** Effects of matrine on intestinal chemokine receptors in mice

Item	Control	1 mg/kg Matrine	5 mg/kg Matrine	10 mg/kg Matrine
Jejunum				
CCR2	1.00 ± 0.13	1.21 ± 0.16	1.26 ± 0.13	1.32 ± 0.12
CCR5	1.00 ± 0.11b	1.09 ± 0.11b	1.17 ± 0.12b	1.43 ± 0.14a
CCR6	1.00 ± 0.07b	1.09 ± 0.16b	1.14 ± 0.13b	1.75 ± 0.18a
CCR7	1.00 ± 0.15b	1.17 ± 0.13b	1.65 ± 0.11a	1.88 ± 0.21a
CCR8	1.00 ± 0.09	1.12 ± 0.16	1.35 ± 0.25	1.43 ± 0.24
Ileum				
CCR2	1.00 ± 0.07b	1.16 ± 0.17b	1.18 ± 0.14b	1.73 ± 0.07a
CCR5	1.00 ± 0.17b	1.19 ± 0.12ab	1.25 ± 0.17ab	1.43 ± 0.14a
CCR6	1.00 ± 0.05	1.19 ± 0.19	1.93 ± 0.19	1.06 ± 0.14
CCR7	1.00 ± 0.08b	1.43 ± 0.13a	1.77 ± 0.18a	2.01 ± 0.25a
CCR8	1.00 ± 0.14	1.15 ± 0.16	1.21 ± 0.14	1.38 ± 0.28

Data are expressed as the mean ± standard error of the mean. Values in the same row with different superscripts are significant (*P <* 0.05), while values with same superscripts are not significant different (*P* > 0.05).

### Matrine alleviates LPS-induced intestinal inflammatory response in mice and Caco-2 cells

LPS was used to induce intestinal inflammation in mice and the results showed that LPS injection markedly caused intestinal inflammatory response evidenced by the increased cytokines (IL-1β, IL-10, IL-17, and TNF-α) (*P <* 0.05) (Table 4). However, dietary 10 mg/kg matrine treatment exhibited an anti-inflammatory function in LPS-challenged mice via reducing intestinal IL-17 expression (*P <* 0.05). Meanwhile, IL-1β in the jejunum and IL-10 in the ileum also tended to be decreased after matrine exposure (*P >* 0.05) (Table 4).

The article "Matrine alleviates lipopolysaccharide-induced intestinal inflammation and oxidative stress via CCR7 signal" was retracted in 2023. Reasons: results that could not be reproduced; unreliable results or conclusions.

**Table 4:** Matrine alleviates LPS-induced intestinal inflammatory response in mice

Item	Control	LPS	LPS + Matrine
Jejunum			
IL-1β	1.00 ± 0.09b	1.64 ± 0.19a	1.36 ± 0.16ab
IL-10	1.00 ± 0.12b	1.43 ± 0.17a	1.52 ± 0.19a
IL-17	1.00 ± 0.08b	1.73 ± 0.21a	1.23 ± 0.15b
TNF-α	1.00 ± 0.14b	1.54 ± 0.15a	1.43 ± 0.09a
Ileum			
IL-1β	1.00 ± 0.07b	1.96 ± 0.18a	1.73 ± 0.18a
IL-10	1.00 ± 0.14b	1.59 ± 0.23a	1.36 ± 0.14ab
IL-17	1.00 ± 0.12b	1.75 ± 0.17a	1.29 ± 0.15b
TNF-α	1.00 ± 0.15	1.35 ± 0.13	1.28 ± 0.15

Data are expressed as the mean ± standard error of the mean. Values in the same row with different superscripts are significant (*P <* 0.05), while values with same superscripts are not significant different (*P* > 0.05).

Caco-2 cells were incubated with different dosages of matrine (0, 0.001, 0.01, 0.1, 0.5, 1, 2 and 5 mM) and LPS (0, 10, 50, 100, and 200 μM) and we selected 0.5 mM matrine and 100 uM LPS for the following analysis according to the cell viability (Figure 1A and 1B). Meanwhile, we found that 0.5 mM matrine treatment markedly alleviated LPS-caused reduction in cell viability (*P <* 0.05) (Figure 1C). We further tested cellular cytokines (i.e. IL-1β, IL-10, IL-17, and TNF-α) after exposure to matrine (Figure 1D–1G) and LPS and the results showed that LPS markedly enhanced cellular IL-1β, IL-10, IL-17, and TNF-α production (*P <* 0.05), while matrine reduced LPS-induced IL-1β and IL-17 generation (*P <* 0.05).

**Figure 1:** Effects of matrine and LPS on cellular viability and inflammatory cytokines Data are expressed as the mean ± standard error of the mean. Values in the same row with different superscripts are significant (*P <* 0.05), while values with same superscripts are not significant different (*P* > 0.05).

### Matrine alleviates LPS-induced intestinal oxidative stress in mice

LPS-challenged mice exhibited a marked oxidative injury evidenced by the decreased ileal SOD and T-AOC activities and higher intestinal MDA level (*P <* 0.05) (Table 5). Matrine treatment significantly decreased jejunal and ileal MDA production (*P <* 0.05), suggesting an antioxidant function in LPS-challenged mice (Table 5).

**Table 5:** Matrine alleviates LPS-induced intestinal oxidative stress in mice

Item	Control	LPS	LPS + Matrine
Jejunum			
SOD U/mgprot	79.23 ± 8.72	71.38 ± 13.64	82.19 ± 12.71
T-AOC U/gprot	0.53 ± 0.06	0.49 ± 0.08	0.43 ± 0.09
MDA uM/mgprot	12.38 ± 1.25b	16.73 ± 1.15a	13.44 ± 1.53b
Ileum			
SOD U/mgprot	71.23 ± 11.53a	56.23 ± 11.38b	61.93 ± 10.29b
T-AOC U/gprot	0.64 ± 0.08a	0.51 ± 0.04b	0.58 ± 0.09ab
MDA uM/mgprot	15.33 ± 1.58b	21.22 ± 2.17a	17.24 ± 1.34b

Data are expressed as the mean ± standard error of the mean. Values in the same row with different superscripts are significant (*P <* 0.05), while values with same superscripts are not significant different (*P* > 0.05).

The article "Matrine alleviates lipopolysaccharide-induced intestinal inflammation and oxidative stress via CCR7 signal" was retracted in 2023. Reasons: results that could not be reproduced; unreliable results or conclusions.

### CCR7 involves in matrine-mediated inflammation and oxidative stress in Caco-2 cells

CCR7 was upregulated in the intestine after dietary supplementation with matrine in mice, thus CCR7 was further determined *in vitro* model after matrine and LPS treatment. The results showed that LPS inhibited cellular CCR7 expression, while matrine enhanced CCR7 protein abundance (*P <* 0.05) (Figure 2A and 2B).

**Figure 2:** Effects of matrine, LPS, and CCR7-siRNA on CCR7 expression and inflammatory cytokines Data are expressed as the mean ± standard error of the mean. Values in the same row with different superscripts are significant (*P <* 0.05), while values with same superscripts are not significant different (P > 0.05).

We further inhibited cellular CCR7 expression via CCR7-siRNA transfection (Figure 2C and 2D) and found that CCR7 inhibition blocked the anti-inflammatory effects of matrine in LPS-challenged cells, evidenced by the enhanced IL-1β, IL-10, IL-17, and TNF-α production (Figure 2E–2H). In addition, CCR7-siRNA transfection exacerbated LPS induced cellular inflammation (*P <* 0.05). These results indicated that CCR7 involved in matrine-mediated inflammatory response in Caco-2 cells.

Cellular SOD and T-AOC activities and MDA level were also tested (Figure 3A–3C) and the results showed that LPS exposure markedly inhibited cellular T-AOC activity and enhanced MDA abundance (*P <* 0.05), suggesting that LPS induced cellular oxidative stress in Caco-2 cells. Matrine enhanced cellular T-AOC activity (*P <* 0.05) but failed to alleviate MDA generation compared with LPS treatment (*P >* 0.05). Meanwhile, CCR7-siRNA transfection blocked the antioxidant function of matrine in LPS-induced oxidative stress and exacerbated LPS-induced oxidative stress (*P <* 0.05).

**Figure 3:** Effects of effects of matrine, LPS, and CCR7-siRNA on oxidative indexes Data are expressed as the mean ± standard error of the mean. Values in the same row with different superscripts are significant (*P <* 0.05), while values with same superscripts are not significant different (*P* > 0.05).

## DISCUSSION

Matrine, a kind of alkaloid component isolated from the roots of Sophora species, has been widely demonstrated to exhibit anti-inflammatory and antioxidant functions in various models [1, 3, 7, 8]. In this study, we found that matrine improved intestinal inflammatory status and antioxidant balance. In LPS-challenged mice and Caco-2 cells, matrine alleviated LPS-induced inflammation and oxidative stress, which might be associated with CCR7 signal.

The article "Matrine alleviates lipopolysaccharide-induced intestinal inflammation and oxidative stress via CCR7 signal" was retracted in 2023. Reasons: results that could not be reproduced; unreliable results or conclusions.

The present study exhibited that dietary matrine improved intestinal inflammatory status via mediating IL-1β and IL-17 expression. After LPS treatment, matrine significantly alleviated LPS-induced IL-1β upregulation. These results indicated that matrine exhibited an anti-inflammatory function, which has been further confirmed by the *in vitro* data. Liu et al. reported that administration of matrine significantly increased serum production of IL-4, IL-5, IL-10, and TGF-β1 in experimental autoimmune encephalomyelitis [9]. In LPS-induced acute lung injury in mice, matrine reduced the production of inflammatory mediators, such as TNF-α, IL-6 and HMGB1, which was possibly associated with inhibition of NF-κB [10]. NF-κB has been considered as one of the key regulators in the immunological and inflammatory setting [11–14] and matrine has been suggested to involves in NF-κB signal to regulate inflammation [15, 16].

Compelling evidences have demonstrated the antioxidant function of matrine via enhancing antioxidant enzymes activities and reducing free radical species [5, 17–20]. In the diabetic cardiomyopathy in rats, the cardiac tissues showed a marked excessive free radical species production, while pretreatment with matrine significantly improved oxidative balance and reduced free radical species [21]. Meanwhile, matrine has been also demonstrated to enhance antioxidant function against progression of high-fructose diet-induced steatohepatitis [17]. Similarly with previous studies, we also found that dietary matrine improved intestinal antioxidant function in mice and alleviated LPS induced oxidative stress in mice and Caco-2 cells via influencing T-AOC and MDA. MDA is a common oxidative product from lipid oxidation [22] and the reduction of MDA in this study suggested an antioxidant function of matrine in LPS-challenged mice and Caco-2 cells. These results further confirmed the antioxidant effect of marine.

Chemokine receptors have been widely investigated in inflammatory response and oxidative stress [23–25]. In this study, we firstly investigated several chemokine receptors after dietary matrine and the results showed that matrine enhanced CCR2, CCR5, CCR6, and CCR7 expressions in mice, especially for CCR7. CCR7 involves in inflammatory and immune response via regulating T-cell homeostasis, T-cell activation and, polarization, which play an important role in the induction and maintenance of chronic inflammation [26–29]. Thus, we further used CCR7-siRNA transfection to inhibit CCR7 expression in Caco-2 cells and found that CCR7-siRNA transfection blocked the anti-inflammatory and antioxidant functions after LPS treatment, suggesting that CCR7 involved in matrine mediated inflammation and oxidative stress. CCR7-knockout mice exhibited greater inflammation and higher release of IL-5, IL-13, TGF-β, and IL-17 compared to wild-type mice [30, 31]. These results provide a novel therapeutic target for inflammatory and oxidative diseases.

The article "Matrine alleviates lipopolysaccharide-induced intestinal inflammation and oxidative stress via CCR7 signal" was retracted in 2023. Reasons: results that could not be reproduced; unreliable results or conclusions.

In conclusion, matrine improved intestinal inflammatory and antioxidant function in mice and Caco-2 cells against LPS exposure. The mechanism might be associated with CCR7 signal, which further regulated inflammatory response and oxidative stress.

## MATERIALS AND METHODS

### Animal model and groups

This study was approved by the animal welfare committee of Shandong Provincial Hospital Affiliated to Shandong University. 40 female Balb/c mice (21.32 ± 2.17 g) were used to investigate the effects of dietary different matrine dosages on inflammatory status. Animals were randomly assigned into 4 groups (*n* = 10) and fed with 4 different matrine diet: 0, 1, 5, and 10 mg/kg matrine for 4 weeks. Then all animals were killed and eye blood and intestine were harvested.

To investigate the effects of matrine on LPS induced-inflammation in mice, 30 female Balb/c mice (20.13 ± 1.65 g) were randomly assigned to daily subcutaneous injections of LPS (25 μg) [32], PBS as a control, and LPS plus dietary 10 mg/kg matrine. After 4 weeks, animals were killed for sample collection.

### Cell culture

Human epithelial Caco-2 cells were grown in Dulbecco's modified Eagle medium (DMEM)/F12 supplemented with 10% FBS (HyClone, Logan, UT) and 50 U/mL penicillin–streptomycin and maintained at 37°C in a humidified chamber of 5% CO_2_. Confluent cells (85–90%) were incubated with different concentrations of matrine (0, 0.001, 0.01, 0.1, 0.5, 1, 2, and 5 mM) and LPS (0, 10, 50, 100, and 200 μM) for 4 days to establish inflammatory model [33].

### CCR7-siRNA transfection

Human CCR7-siRNA was obtained from Guangzhou RiboBio and the sequences were accorded to a previous report [34]. Cells were cultured in 6-well plates and grown to 30–50% confluence before transfection. The duplexes were diluted to give a final concentration of 30 nM. The siRNA was transfected into cells using Lipofectamine RNAiMAX reagent according to the manufacturer's instructions (Invitrogen).

### Measurement of oxidative stress

Intestinal and cell SOD and T-AOC activity were measured using spectrophotometric kits (Nanjing Jiangcheng Biotechnology Institute, China). MDA levels were measured using a thiobarbituric acid reactive substances assay kit according to the manufacturer's instructions (Nanjing Jiangcheng Biotechnology Institute, China). IL-1β, IL-10, IL-17, and TNF-α were measured using ELISA kits (CUSABIO, Wuhan, China).

The article "Matrine alleviates lipopolysaccharide-induced intestinal inflammation and oxidative stress via CCR7 signal" was retracted in 2023. Reasons: results that could not be reproduced; unreliable results or conclusions.

### Real-time PCR

One piece of jejunum, ileum, and ileum were harvested and stored at −80 °C. Total RNA of these tissues was isolated with TRIZOL regent (Invitrogen, USA) and reverse transcribed into the first strand (cDNA) using DNase I, oligo (dT) 20 and Superscript II reverse transcriptase (Invitrogen, USA). The reverse transcription was conducted at 37°C for 15 min, 95°C 5 sec. Primers were designed with Primer 5.0 according to the gene sequence of mouse to produce an amplification product (Table 6). β-actin was chosen as the house-keeping gene to normalize target gene levels. The PCR cycling condition was 36 cycles at 94°C for 40 sec, 60°C for 30 sec and 72°C for 35 sec. The relative expression was expressed as a ratio of the target gene to the control gene using the formula 2^–(ΔΔCt)^, where ΔΔCt = (Ct_Target_–Ct_β-actin_)_treatment_–(Ct_Target_–Ct_β-actin_)_control_. Relative expression was normalized and expressed as a ratio to the expression in the control group.

**Table 6:** Primers used in this study

Genes	No.	Nucleotide sequence of primers (5′–3′)	bp
*β-Actin*	NM_007393.5	F: CCACCATGTACCCAGGCATTR: AGGGTGTAAAACGCAGCTCA	253
IL-1β	NM_008361.4	F: TGCCACCTTTTGACAGTGATGR: AAGGTCCACGGGAAAGACAC	220
IL-10	NM_010548.2	F: TAAGGCTGGCCACACTTGAGR: GTTTTCAGGGATGAAGCGGC	209
*IL-17*	NM_010552.3	F: GCTGACCCCTAAGAAACCCCR: GAAGCAGTTTGGGACCCCTT	162
*TNF-α*	NM_013693.3	F: ATGGCCTCCCTCTCATCAGTR:TTTGCTACGACGTGGGCTAC	*97*
*CCR2*	NM_009915.2	F: GCCATCATAAAGGAGCCATACCR: ATGCCGTGGATGAACTGAGG	*173*
*CCR5*	NM_009917.5	F: GTTGTTTTGGAGAACGCCCCR: CAACACTGCTCCGAAACTGC	*187*
CCR6	NM_009835.4	F: ATACACAAGGCACCGCTTGAR: GGCAGACACTCACAGTACCC	283
CCR7	NM_007719.2	F: GGAAACCCAGGAAAAACGTGCR: TCCTTCTTGAAGCACACCGA	145
CCR8	NM_007720.2	F: TCTGGGTCCCATTCAACGTGR: AGATGTGGCTGCAGCTCTTT	219

F: forward; R: reverse.

### Western bolt for CCR7 expression

One piece of jejunum, ileum, and ileum were harvested and stored at –80°C. Proteins were extracted with using protein extraction reagents (Thermo Fisher Scientific Inc., USA) and the concentration was tested using BCA protein assay (Sigma-Aldrich, USA). Proteins (30 μg) were separated by SDS–polyacrylamide gel electrophoresis and electrophoretically transferred to a polyvinylidene difluoride (PVDF) membrane (BioRad, Hercules, CA, USA). Membranes were blocked and then incubated with the following primary antibodies: Anti-CCR7 antibody [Y59] (ab32527) (Abcam). Mouse β–actin antibody (Sigma) was used for protein loading control. After primary antibody incubation, membranes were washed, incubated with alkaline phosphatase-conjugated anti-mouse or anti-rabbit IgG antibodies (Promega, Madison, WI, USA), and quantified and digitally analyzed using the image J program (NIH).

The article "Matrine alleviates lipopolysaccharide-induced intestinal inflammation and oxidative stress via CCR7 signal" was retracted in 2023. Reasons: results that could not be reproduced; unreliable results or conclusions.

### Statistical analysis

All data were analyzed by SPSS 17.0 software. Difference was tested by Ducan's multiple comparison test. Data are expressed as the mean ± SEN. Values in the same row with different superscripts are significant (*P <* 0.05).
